The article "Optimized multiple-attribute group decision-making through employing probabilistic hesitant fuzzy TODIM and EDAS technique and application to teaching quality evaluation of international Chinese course in higher vocational colleges" was retracted in 2025. Reasons: unreliable results or conclusions; concerns about the peer review; concerns about the citations.

# Optimized multiple-attribute group decision-making through employing probabilistic hesitant fuzzy TODIM and EDAS technique and application to teaching quality evaluation of international Chinese course in higher vocational colleges

**DOI:** 10.1016/j.heliyon.2024.e25758

**Published:** 2024-02-10

**Authors:** Fangfang Xia

**Affiliations:** School of International Education, Yiwu Industrial & Commercial College, Yiwu, 322000, Zhejiang, China

**Keywords:** Multiple-attributes group decision-making (MAGDM), Probabilistic hesitant fuzzy sets (PHFSs), TODIM technique, EDAS technique, Teaching quality evaluation

## Abstract

With the construction and development of the “the Belt and Road”, the international community has an increasing demand for high-quality technical and skilled talents who both understand Chinese and have an international perspective. Exploring a Chinese curriculum system suitable for the development of international students is conducive to promoting the international development of vocational education, improving the quality of international student training, providing talent support for Chinese and foreign enterprises, and promoting the “going out” of Chinese enterprises and international production capacity cooperation. The training of international students in higher vocational colleges starts late, has little experience, lacks theoretical innovation, and lacks the development characteristics of vocational education. The teaching quality evaluation of international Chinese course in higher vocational colleges is multiple-attributes group decision-making (MAGDM). Recently, the TODIM and EDAS technique has been employed to manage MAGDM. The probabilistic hesitant fuzzy sets (PHFSs) are employed as a useful tool for depicting uncertain information during the teaching quality evaluation of international Chinese course in higher vocational colleges. In this paper, the probabilistic hesitant fuzzy TODIM-EDAS (PHF-TODIM-EDAS) technique is built to manage the MAGDM under PHFSs. Finally, the numerical example for teaching quality evaluation of international Chinese course in higher vocational colleges is employed to show the PHF-TODIM-EDAS technique. The main contribution of this paper is outlined: (1) the TODIM technique based on EDAS technique has been extended to PHFSs based on CRITIC technique; (2) the CRITIC technique is employed to derive weight numbers under PHFSs. (3) the PHF-TODIM-EDAS technique is founded to manage the MAGDM under PHFSs; (4) a numerical case study for teaching quality evaluation of international Chinese course in higher vocational colleges and some comparative analysis is supplied to validate the proposed PHF-TODIM-EDAS technique.

## 1 Introduction

For a long time, countries and universities have invested a lot of resources in the teaching of international Chinese courses for international students, and have achieved certain results, but there are also certain problems [1]. Because the basic Chinese knowledge of foreign students is very weak, and even a considerable number of foreign students' Chinese level is zero, in this case, teachers will pay more attention to the teaching of basic Chinese knowledge. Therefore, many colleges and universities tend to pay more attention to the training of basic skills of Chinese language, that is, listening, speaking, reading and writing, while ignoring the vocational technology and skill education based on Chinese [2]. This way of learning language knowledge, without access to professional knowledge, is not only easy to make foreign students feel “tired” in learning, but also not conducive to the stimulation of foreign students' enthusiasm for learning. So after realizing basic Chinese communication, we found a problem limited by professional Chinese knowledge, foreign students have some difficulties in professional learning, and domestic vocational colleges also lack relevant professional Chinese teaching experience, so the connection between basic Chinese and professional Chinese is not smooth [3]. Specifically, it includes four aspects: First, there is a bias in the cognition of the teaching of international Chinese courses. The basic knowledge of Chinese language is important for foreign students, but the learning of language knowledge cannot be taken as the whole. Relevant corporate cultural knowledge, corporate management knowledge, technical skills and standards are also essential, which is the key to cultivating the “cultural and technological talents” that are in short supply in countries along the “the Belt and Road” [4]. Second, the assessment form of international Chinese course is single. The result of the Chinese proficiency test has become the standard to measure the level of Chinese proficiency, which violates its language characteristics. It is a question that needs to be considered and solved whether we can combine the course certificate assessment and establish the grade test standard of professional Chinese as the reference basis for the selection and evaluation of local technical and skilled talents of overseas students and overseas Chinese-funded enterprises. Third, the integration of Chinese language learning and technical skills learning is relatively low. Any learning cannot be separated from the creation of a good learning environment [5]. A single environment in the classroom can neither provide a realistic situation for students' communication, nor enable students to link language knowledge with professional learning, because book knowledge can realize its application value only when combined with practice. How to create a good environment, learn Chinese language in an immersive environment, and carry out listening, speaking, reading and writing training; To enable foreign students to apply Chinese in the practical environment and complete the communication and practical tasks in the workplace is another issue that needs to be considered [6]. Fourth, the curriculum content is not reasonable enough to meet the diverse needs of international students. Generally speaking, there are two conditions for foreign students to study in a country. One is to learn the language and culture of the country; The second is to learn technical skills in relevant professional fields with the help of language knowledge and cultural knowledge on the basis of mastering the Chinese language [7]. The group of overseas students from countries along the “the Belt and Road” is more the second case. However, at present, international Chinese courses for foreign students in China are mainly Chinese conversation, Chinese listening, Chinese reading and writing, and Chinese synthesis, and HSK (hàn yǔ shuǐ píng kǎo shì) three-level counseling is also offered. Whether students pass the HSK Level III exam has an important impact on whether they can directly enter the relevant professional courses. The combination of international Chinese course teaching and vocational skills is not high, and there is a lack of necessary transition between basic Chinese knowledge and professional knowledge.

In real life, many phenomena and events are complex and diverse, but they can be divided into definite and uncertain ones [[8], [9], [10], [11]]. Correspondingly, certain phenomena are called deterministic mathematics, where the determined criteria divide their phenomena into well-defined classes, such as natural laws, precision phenomena, etc [[12], [13], [14]]. The laws are certain and can be followed. For example, in classical set theory, the membership relationship between elements and sets within a given range must be clear, or “belong to”, Either “does not belong”, usually represented by “0″ or “1″ to indicate this degree of membership [[15], [16], [17]]. Both must be in one place, and only in one place, satisfying the law of exclusion. Therefore, classical set theory only describes the phenomenon of “either this or that” with clear extensions, while concepts and phenomena with unclear extensions cannot be accurately and reasonably represented [[18], [19], [20]]. However, due to the complexity of social phenomena, the vast majority of phenomena and events are uncertain. As the number of participants in decision-making increases, the decision-making process becomes more complex [[21], [22], [23], [24]]. Therefore, multi-attribute group decision-making (MAGDM) has developed into an extremely important research field in modern decision-making theory and decision-making science, and has been widely applied in many fields such as engineering, logistics, medicine, and military [[25], [26], [27], [28], [29]]. Since Zadeh [30] proposed the theory of fuzzy sets (FSs) in 1965, this theory has been commonly used to deal with problems with fuzziness and uncertainty in real life. Atanassov [31] defined intuitionistic fuzzy sets (IFSs), which believe that the sum of membership and non-membership should be less than or equal to 1. The Pythagorean fuzzy sets (PFSs) proposed by Yager [32] expanded the range of membership and non-membership to a sum of squares less than or equal to 1. Considering that decision-makers may hesitate about membership values during the decision-making process, Torra [33] proposed Hesitant fuzzy sets (HFSs). In recent years, scholars both domestically and internationally have conducted extensive research on HFSs [[34], [35], [36]]. Zhu, Xu and Xia [37] proposed dual hesitant fuzzy sets (DHFSs) by defining possible membership and possible non-membership. Xu and Zhou [38] proposed probabilistic hesitant fuzzy sets (PHFSs) based on hesitant fuzzy sets, which not only provide all the membership degrees of each evaluation scheme, but also provide the probability corresponding to each membership degree. The teaching quality evaluation of international Chinese course in higher vocational colleges can be regarded as a MAGDM. The probabilistic hesitant fuzzy sets (PHFSs) [38] are employed as a tool for portraying uncertain information during the teaching quality evaluation of international Chinese course in higher vocational colleges. Furthermore, compared with other decision techniques [[39], [40], [41], [42], [43]], many studies employed the traditional TODIM technique [[44], [45], [46]] and EDAS technique [47,48] separately to obtain the most optimal decision choice. Until now, no or few techniques have been investigated on CRITIC technique [49] and TODIM technique [44] based on EDAS technique [47,48] under PHFSs. Therefore, an integrated probabilistic hesitant fuzzy TODIM-EDAS (PHF-TODIM-EDAS) technique is constructed to manage MAGDM under PHFSs. An illustrative example for teaching quality evaluation of international Chinese course in higher vocational colleges and some comparative analysis is constructed to demonstrate the validity and reliability of PHF-TODIM-EDAS technique. The main aim and motivation of this paper is outlined: (1) the TODIM technique based on EDAS technique has been extended to PHFSs based on CRITIC technique; (2) the CRITIC technique is employed to derive weight numbers under PHFSs. (3) the PHF-TODIM-EDAS technique is founded to manage the MAGDM under PHFSs; (4) a numerical case study for teaching quality evaluation of international Chinese course in higher vocational colleges and some comparative analysis is supplied to verify the proposed PHF-TODIM-EDAS technique. Thus, the main advantages of the proposed PHF-TODIM-EDAS technique are outlined: (1) the proposed PHF-TODIM-EDAS technique not only handles the bounded rationality in real MADM issues, but also portrays the hamming distances from the PHFNAS. (2) the proposed PHF-TODIM-EDAS technique analyze the behavior of the TODIM technique and EDAS technique as MADM when they are hybridized. The main disadvantages of the proposed PHF-TODIM-EDAS technique fails to manage the consensus theory and regret theory in the proposed MAGDM.

The research structure of this paper is constructed. In Sect. 2, the PHFSs is fully introduced. In Sect. 3, PHF-TODIM-EDAS technique is put forward under PHFSs. Sect. 4 gives the study example for teaching quality evaluation of international Chinese course in higher vocational colleges and some comparative decision analysis. Some remarks are constructed in Sect. 5.

## 2 Preliminaries

Xu and Zhou [38] put forward the PHFSs based on the HFSs [33,[50], [51], [52], [53], [54]].

Definition 1 [38]. Let θ be a fixed collection, a PHFSs on Θ is managed in Eq. (1):

(1) $$VH=\left\{<\theta ,vh_{\theta }\left(vp_{\theta }\right)>|\theta \in \Theta \right\}$$

where $vh_{\theta }\left(vp_{\theta }\right)$ is a set of numbers, and $vh_{\theta }\left(vp_{\theta }\right)\in \left[0,1\right]$ denoting the possible membership of the element θ∈Θ to the set Θ, $vh_{\theta }$ is called a hesitant fuzzy number (HFN), $vp_{\theta }$ is a group of probabilities connected with $vh_{\theta }$.

For convenience, vh(vp) is called a probabilistic hesitant fuzzy number (PHFN), and the set of all PHFEs are constructed as $vh\left(vp\right)=\left\{vh^{\left(v\varphi \right)}\left(vp^{\left(v\varphi \right)}\right)|\;v\varphi =1,2,\cdots ,\#vh\left(vp\right)\right\}$, where $vp^{\left(v\varphi \right)}$ is the probability numbers of the $vh^{\left(v\varphi \right)}$, #vh(vp) is the number of membership, and $\sum_{v\varphi =1}^{\#vh\left(vp\right)}vp^{\left(v\varphi \right)}=1$.

Definition 2 [38]. $vh_{1}\left(vp\right)=\left\{vh_{1}^{\left(v\varphi \right)}\left(vp_{1}^{\left(v\varphi \right)}\right)|\;v\varphi =1,2,\cdots ,\#vh_{1}\left(vp\right)\right\}$ and $vh_{2}\left(vp\right)=\left\{vh_{2}^{\left(v\varphi \right)}\left(vp_{2}^{\left(v\varphi \right)}\right)|\;v\varphi =1,2,\cdots ,\#vh_{2}\left(vp\right)\right\}$ be two PHFSs, $\#vh_{1}\left(vp\right)$ and $\#vh_{2}\left(vp\right)$ are the length of $vh_{1}\left(vp\right)$ and $vh_{2}\left(vp\right)$. If $\#vh_{1}\left(vp\right)>\#vh_{2}\left(vp\right)$, then add $\#vh_{1}\left(vp\right)-\#vh_{2}\left(vp\right)$ HFNs to $vh_{2}\left(vp\right)$. The added HFNs are the smallest HFNs in $vh_{2}\left(vp\right)$ and the probabilities are zero.

Definition 3 [38]. For the $vh_{1}\left(vp\right)=\left\{vh_{1}^{\left(v\varphi \right)}\left(vp_{1}^{\left(v\varphi \right)}\right)|\;v\varphi =1,2,\cdots ,\#vh_{1}\left(vp\right)\right\}$, the expected numbers $EV\left(vh_{1}\left(vp\right)\right)$ and deviation degree $DD\left(vh_{1}\left(vp\right)\right)$ is constructed in Eq. (2)- Eq. (3):

(2) $$EV\left(vh_{1}\left(vp\right)\right)=\sum_{v\varphi =1}^{\#vh_{1}\left(vp\right)}\left(vh_{1}^{\left(v\varphi \right)}\times vp_{1}^{\left(v\varphi \right)}\right)$$

(3) $$DD\left(vh_{1}\left(vp\right)\right)=\sqrt{\sum_{v\varphi =1}^{\#vh_{1}\left(vp\right)}{\left(vh_{1}^{\left(v\varphi \right)}\times vp_{1}^{\left(v\varphi \right)}-EV\left(vh_{1}\left(vp\right)\right)\right)}^{2}}$$

By Eqs. (2), (3), the order for two PHFEs is constructed: (1) if $EV\left(vh_{1}\left(vp\right)\right)>EV\left(vh_{2}\left(vp\right)\right)$, $vh_{1}\left(vp\right)>vh_{2}\left(vp\right)$; (2)if $EV\left(vh_{1}\left(vp\right)\right)=EV\left(vh_{2}\left(vp\right)\right)$, if $DD\left(vh_{1}\left(vp\right)\right)=DD\left(vh_{2}\left(vp\right)\right)$, then $vh_{1}\left(vp\right)=vh_{2}\left(vp\right)$; if $DD\left(vh_{1}\left(vp\right)\right)<DD\left(vh_{2}\left(vp\right)\right)$, then, $vh_{1}\left(vp\right)>vh_{2}\left(vp\right)$.

Definition 4 [38]. Let $vh_{1}\left(vp\right)=\left\{vh_{1}^{\left(v\varphi \right)}\left(vp_{1}^{\left(v\varphi \right)}\right)|\;v\varphi =1,2,\cdots ,\#vh_{1}\left(vp\right)\right\}$ and $vh_{2}\left(vp\right)=\left\{vh_{2}^{\left(v\varphi \right)}\left(vp_{2}^{\left(v\varphi \right)}\right)|\;v\varphi =1,2,\cdots ,\#vh_{2}\left(vp\right)\right\}$ with $\#vh_{1}\left(vp\right)=\#vh_{2}\left(vp\right)=\#vh\left(vp\right)$, then Hamming distance $HD\left(vh_{1}\left(vp\right),vh_{2}\left(vp\right)\right)$ is managed in Eq. (4):

(4) $$HD\left(vh_{1}\left(vp\right),vh_{2}\left(vp\right)\right)=\frac{\sum_{v\varphi =1}^{\#vh\left(vp\right)}\left|vh_{1}^{\left(v\varphi \right)}\times vp_{1}^{\left(v\varphi \right)}-vh_{2}^{\left(v\varphi \right)}\times vp_{2}^{\left(v\varphi \right)}\right|}{\#vh\left(vp\right)}$$

## 3 The PHF-TODIM-EDAS technique for MADM under PHFSs

Then, PHF-TODIM-EDAS technique is built to manage the MADM, where the decision-making information are depicted through PHFSs. Let $VL=\left\{VL_{1},VL_{2},\cdots ,VL_{m}\right\}$ be alternatives and $VT=\left\{VT_{1},VT_{2},\cdots ,VT_{n}\right\}$ be attributes with weight information $vw=\left(vw_{1},vw_{2},\cdots ,vw_{n}\right)$, where $vw_{j}\in \left[0,1\right]$, $\sum_{j=1}^{n}vw_{j}=1$. Suppose that decision information is denoted as PHFSs $h_{ij}\left(vp\right)=\left\{vh_{ij}^{\left(v\varphi \right)}\left(vp_{ij}^{\left(v\varphi \right)}\right)|\;v\varphi =1,2,\cdots ,\#vh_{ij}\left(vp\right)\right\}\left(i=1,2,\cdots ,m,j=1,2,\cdots ,n\right)$ .

Then, PHF-TODIM-EDAS technique is constructed to manage the MADM issues under PHFSs and CRITIC weight. The detailed algorithms are managed (See Fig. 1).

Stage 1 Obtain the MADM information with PHFSs

Step 1 Found the PHF-matrix $VH={\left[vh_{ij}\left(vp\right)\right]}_{m\times n}$ in Eq. (5)- Eq. (6):

(5) $$\begin{array}{l} \begin{array}{cccc} \;VT_{1} & \;VT_{2}\; & \ldots & \;VT_{n} \end{array}\\ VH={\left[vh_{ij}\left(vp\right)\right]}_{m\times n}=\begin{array}{c} VL_{1}\\ VL_{2}\\ \vdots \\ VL_{m} \end{array}\left[\begin{array}{cccc} vh_{11}\left(vp\right) & vh_{12}\left(vp\right) & \ldots & vh_{1n}\left(vp\right)\\ vh_{21}\left(vp\right) & vh_{22}\left(vp\right) & \ldots & vh_{2n}\left(vp\right)\\ \vdots & \vdots & \vdots & \vdots \\ vh_{m1}\left(vp\right) & vh_{m2}\left(vp\right) & \ldots & vh_{mn}\left(vp\right) \end{array}\right] \end{array}$$

(6) $$VH={\left[vh_{ij}\left(vp\right)\right]}_{m\times n}=\left\{vh_{ij}^{\left(v\varphi \right)}\left(vp_{ij}^{\left(v\varphi \right)}\right)|\;v\varphi =1,2,\cdots ,\#vh_{ij}\left(vp\right)\right\}$$

Step 2 Standardize the $VH={\left[vh_{ij}\left(vp\right)\right]}_{m\times n}$ into $NVH={\left[nvh_{ij}\left(nvp\right)\right]}_{m\times n}$ in Eq. (7)- Eq. (8):

(7) $$\left\{ \begin{array}{cc} nvh_{ij}\left(nvp\right)=vh_{ij}^{\left(v\varphi \right)}\left(vp_{ij}^{\left(v\varphi \right)}\right) & \text{when}\;\text{the}\;\text{decision}\;\text{attribute}\;\text{is}\;\text{positive}\;\\ nvh_{ij}\left(nvp\right)=\left\{1-vh_{ij}^{\left(v\varphi \right)}\left(vp_{ij}^{\left(v\varphi \right)}\right)\right\} & \text{when}\;\text{the}\;\text{decision}\;\text{attribute}\;\text{is}\;\text{negative}\; \end{array}\right.$$

(8) $$NVH={\left[nvh_{ij}\left(nvp\right)\right]}_{m\times n}=\left\{nvh_{ij}^{\left(v\varphi \right)}\left(nvp_{ij}^{\left(v\varphi \right)}\right)|\;v\varphi =1,2,\cdots ,\#nvh_{ij}\left(nvp\right)\right\}$$

Stage 2 Manage the attributes weight numbers through employing CRITIC technique.

Step 3 Implement the attributes weight through employing the CRITIC technique.

The CRITIC technique was put up by Ref. [55], was employed to manage the attributes weight numbers. The computing procedures of the CRITIC technique are managed [56].

(1) Manage the PHFN correlation coefficient $PHFNCC={\left(PHFNCC_{jt}\right)}_{n\times n}$ in Eq. (9).

$$PHFNCC_{jt}=\frac{\sum_{i=1}^{m}\left(\begin{array}{l} \left(\sum_{v\varphi =1}^{\#nvh_{ij}\left(nvp\right)}\left(nvh_{ij}^{\left(v\varphi \right)}\times nvp_{ij}^{\left(v\varphi \right)}\right)-\left(\sum_{v\varphi =1}^{\#nvh_{i}\left(nvp\right)}\left(nvh_{j}^{\left(v\varphi \right)}\times nvp_{j}^{\left(v\varphi \right)}\right)\right)\right)\cdot \\ \left(\sum_{v\varphi =1}^{\#nvh_{it}\left(nvp\right)}\left(nvh_{it}^{\left(v\varphi \right)}\times nvp_{it}^{\left(v\varphi \right)}\right)-\left(\sum_{v\varphi =1}^{\#nvh_{t}\left(nvp\right)}\left(nvh_{t}^{\left(v\varphi \right)}\times nvp_{t}^{\left(v\varphi \right)}\right)\right)\right) \end{array}\right)}{\begin{array}{l} \sqrt{\sum_{i=1}^{m}{\left(\sum_{v\varphi =1}^{\#nvh_{ij}\left(nvp\right)}\left(nvh_{ij}^{\left(v\varphi \right)}\times nvp_{ij}^{\left(v\varphi \right)}\right)-\left(\sum_{v\varphi =1}^{\#nvh_{i}\left(nvp\right)}\left(nvh_{j}^{\left(v\varphi \right)}\times nvp_{j}^{\left(v\varphi \right)}\right)\right)\right)}^{2}}\cdot \\ \sqrt{\sum_{i=1}^{m}{\left(\sum_{v\varphi =1}^{\#nvh_{it}\left(nvp\right)}\left(nvh_{it}^{\left(v\varphi \right)}\times nvp_{it}^{\left(v\varphi \right)}\right)-\left(\sum_{v\varphi =1}^{\#nvh_{t}\left(nvp\right)}\left(nvh_{t}^{\left(v\varphi \right)}\times nvp_{t}^{\left(v\varphi \right)}\right)\right)\right)}^{2}} \end{array}}\text{,}$$

(9) j,t=1,2,…,n

where $nvh_{j}^{\left(v\varphi \right)}\left(nvp_{j}^{\left(v\varphi \right)}\right)=\frac{\sum_{i=1}^{m}nvh_{ij}^{\left(v\varphi \right)}}{m}\left(\frac{\sum_{i=1}^{m}nvp_{ij}^{\left(v\varphi \right)}}{m}\right)$ and $nvh_{t}^{\left(v\varphi \right)}\left(nvp_{t}^{\left(v\varphi \right)}\right)=\frac{\sum_{i=1}^{m}nvh_{it}^{\left(v\varphi \right)}}{m}\left(\frac{\sum_{i=1}^{m}nvp_{it}^{\left(v\varphi \right)}}{m}\right)$.

(2) Manage the PHFN standard deviation numbers (PHFNSDV) in Eq. (10)- Eq. (11).

(10) $$PHFNSDV_{j}=\sqrt{\frac{1}{m}\sum_{i=1}^{m}{\left(\begin{array}{l} \left(\sum_{v\varphi =1}^{\#nvh_{ij}\left(nvp\right)}\left(nvh_{ij}^{\left(v\varphi \right)}\times nvp_{ij}^{\left(v\varphi \right)}\right)\right)\\ -\left(\sum_{v\varphi =1}^{\#nvh_{i}\left(nvp\right)}\left(nvh_{J}^{\left(v\varphi \right)}\times nvp_{J}^{\left(v\varphi \right)}\right)\right) \end{array}\right)}^{2}},j=1,2,\ldots ,n\text{,}$$

(3) Manage the weights numbers of attribute.

(11) $$vw_{j}=\frac{PHFNSDV_{j}\sum_{t=1}^{n}\left(1-PHFNCDC_{jt}\right)}{\sum_{j=1}^{n}\left(PHFNSDV_{j}\sum_{t=1}^{n}\left(1-PHFNCDC_{jt}\right)\right)},j=1,2\ldots ,n\text{,}$$

Stage 3 PHF-TODIM-EDAS technique for MADM

The PHF-TODIM-EDAS technique is managed for MADM issue.

Step 4 Manage relative weight information of $VT_{j}$ as in Eq. (12):

(12) $$rvw_{j}=vw_{j}/\max_{j}vw_{j}\text{,}$$

Step 5 The PHFN dominance degree (PHFNDD) $PHFNDD_{j}\left(VL_{i},VL_{t}\right)$ of $VL_{i}$ over $VL_{t}$ for $VT_{j}$ is constructed in Eq. (13):

(13) $$PHFNDD_{j}\left(VL_{i},VL_{t}\right)=\left\{ \begin{array}{cc} \frac{rvw_{j}\times \sqrt{\left(HD\left(\left(nvh_{ij}\left(nvp\right)\right),\left(nvh_{tj}\left(nvp\right)\right)\right)\right)}}{\sum_{j=1}^{n}rvw_{j}} & \text{if}\;SV\left(nvh_{ij}\left(nvp\right)\right)>SV\left(nvh_{tj}\left(nvp\right)\right)\\ 0 & \text{if}\;SV\left(nvh_{ij}\left(nvp\right)\right)=SV\left(nvh_{tj}\left(nvp\right)\right)\\ -\frac{1}{v\theta }\frac{\sum_{j=1}^{n}rvw_{j}\times \sqrt{\left(HD\left(\left(nvh_{ij}\left(nvp\right)\right),\left(nvh_{tj}\left(nvp\right)\right)\right)\right)}}{rvw_{j}} & \text{if}\;SV\left(nvh_{ij}\left(nvp\right)\right)<SV\left(nvh_{tj}\left(nvp\right)\right) \end{array}\right.$$

The vθ is constructed in line with Ref. [57].

The $PHFNDD_{j}\left(VL_{i},VL_{t}\right)$ with respect to $VT_{j}$ is managed in Eq. (14):

(14) $$\begin{array}{l} PHFNDD_{j}\left(VL_{i}\right)={\left[PHFNDD_{j}\left(VL_{i},VL_{t}\right)\right]}_{m\times m}\\ \begin{array}{cccc} \;VL_{1} & \;VL_{2} & \cdots & \;VL_{m} \end{array}\\ \;=\begin{array}{c} VL_{1}\\ VL_{2}\\ \vdots \\ VL_{m} \end{array}\left[\begin{array}{cccc} 0 & PHFNDD_{j}\left(VL_{1},VL_{2}\right) & \cdots & PHFNDD_{j}\left(VL_{1},VL_{m}\right)\\ PHFNDD_{j}\left(VL_{2},VL_{1}\right) & 0 & \cdots & PHFNDD_{j}\left(VL_{2},VL_{m}\right)\\ \vdots & \vdots & \cdots & \vdots \\ PHFNDD_{j}\left(VL_{m},VL_{1}\right) & PHFNDD_{j}\left(VL_{m},VL_{2}\right) & \cdots & 0 \end{array}\right] \end{array}$$

The overall PHFNDD of $VL_{i}$ over other alternatives for $VT_{j}$ is constructed in Eq. (15):

(15) $$PHFNDD_{j}\left(VL_{i}\right)=\sum_{t=1}^{m}PHFNDD_{j}\left(VL_{i},VL_{t}\right)$$

Then, the overall PHFNDD is managed in Eq. (16):

(16) $$PHFNDD={\left(PHFNDD_{ij}\right)}_{m\times n}=\left[\begin{array}{ccccc} & VT_{1} & VT_{2} & \ldots & VT_{n}\\ VL_{1} & \sum_{t=1}^{m}PHFNDD_{1}\left(VL_{1},VL_{t}\right) & \sum_{t=1}^{m}PHFNDD_{2}\left(VL_{1},VL_{t}\right) & \ldots & \sum_{t=1}^{m}PHFNDD_{n}\left(VL_{1},VL_{t}\right)\\ VL_{2} & \sum_{t=1}^{m}PHFNDD_{1}\left(VL_{2},VL_{t}\right) & \sum_{t=1}^{m}PHFNDD_{2}\left(VL_{2},VL_{t}\right) & \ldots & \sum_{t=1}^{m}PHFNDD_{n}\left(VL_{2},VL_{t}\right)\\ \vdots & \vdots & \vdots & \vdots & \vdots \\ VL_{m} & \sum_{t=1}^{m}PHFNDD_{1}\left(VL_{m},VL_{t}\right) & \sum_{t=1}^{m}PHFNDD_{2}\left(VL_{m},VL_{t}\right) & \ldots & \sum_{t=1}^{m}PHFNDD_{n}\left(VL_{m},VL_{t}\right) \end{array}\right]$$

Step 6 Implement the PHFN average solution (PHFNAS) for attributes in Eq. (17)- Eq. (19).

(17) $$PHFNAS={\left[PHFNAS_{j}\right]}_{1\times n}={\left[\frac{\sum_{i=1}^{m}NPHFNDD_{ij}}{m}\right]}_{1\times n}$$

(18) $$NPHFNDD_{ij}=\frac{PHFNDD_{ij}-PHFNNIS_{j}}{PHFNPIS_{j}-PHFNNIS_{j}}\text{,}$$

(19) $$PHFNPIS_{j}=\max_{j=1}^{n}PHFNDD_{ij},PHFNNIS_{j}=\min_{j=1}^{n}PHFNDD_{ij}$$

Step 7 Implement the PHFN positive distance from average (PHFNPDA) and PHFN negative distance from average (PHFNNDA) in Eq. (20)- Eq. (21):

(20) $$PHFNPDA_{ij}={\left[PHFNPDA_{ij}\right]}_{m\times n}=\frac{\max\left(0,\left(NPHFNDD_{ij}-PHFNAS_{j}\right)\right)}{PHFNAS_{j}}\text{,}$$

(21) $$PHFNNDA_{ij}={\left[PHFNNDA_{ij}\right]}_{m\times n}=\frac{\max\left(0,\left(PHFNAS_{j}-NPHFNDD_{ij}\right)\right)}{PHFNAS_{j}}\text{,}$$

Step 8 Implement the $PHFNSP_{i}$ and $PHFNSN_{i}$ in Eq. (22)- Eq. (23).

(22) $$PHFNSP_{i}=\sum_{j=1}^{n}vw_{j}\cdot PHFNPDA_{ij},PHFNSN_{i}=\sum_{j=1}^{n}vw_{j}\cdot PHFNNDA_{ij}\text{,}$$

Step 9 Normalized the $PHFNSP_{i}$ and $PHFNSN_{i}$:

(23) $$PHFNNSP_{i}=\frac{PHFNSP_{i}}{\max_{i}\left(PHFNSP_{i}\right)},PHFNNSN_{i}=1-\frac{PHFNSN_{i}}{\max_{i}\left(PHFNSN_{i}\right)}\text{,}$$

Step 10 Implement the PHFN appraisal numbers (PHFNAV) for decision alternative in Eq. (24).

(24) $$PHFNAV_{i}=\frac{1}{2}\left(PHFNNSP+PHFNNSN_{i}\right)$$

Step 11 In line with PHFNAV, the higher PHFNAV is the optimal choice.

**Fig. 1:** The steps of PHF-TODIM-EDAS technique for MADM under PHFSs.

## 4 Numerical example and comparative analysis

### 4.1 Numerical example for teaching quality evaluation of international Chinese course

After several years of exploration and practice, the teaching of Chinese as a foreign language in the context of “Chinese+" has achieved some experience and results, but how to further improve the teaching content of “Chinese+" and build a more scientific and reasonable curriculum system still needs to be further considered and summarized in practice. The advantages of international Chinese education and vocational education should be fully considered, and the teaching content and teaching methods should always be set according to the needs of learners, industry enterprises and regional economic development. At the same time, we should adhere to the employment-oriented principle and organically combine the communicative and practical nature of language teaching with the professional and practical nature of skill teaching. To change the current situation of traditional language teachers' lack of professional skills and the relatively weak language ability of professional teachers, and to cultivate the “Chinese+" teachers with both language teaching ability and practical skills is the key to promote the rapid development of “Chinese+". So far, there are mainly the following problems: (1) The problem of “marginalization” of Chinese courses for international students in higher vocational colleges. Generally speaking, many higher vocational colleges start late in training international students and lack experience. Therefore, it is necessary to distinguish between primary and secondary, reasonably allocate the proportion of professional and Chinese courses, do a good job of synchronous connection between professional courses and Chinese courses, strengthen the discussion and interaction between teachers, and better integrate Chinese courses into the training of technical and skilled personnel. (2) The relationship between Chinese language teaching and HSK test for international students HSK test is the requirement for international students to enter and graduate, which has great attraction for international students. However, Chinese language teaching is not only to deal with HSK test, but also to improve international students' Chinese language application ability and professional skills. Therefore, in the construction of the Chinese curriculum system for international students, the HSK test cannot be taken as the key to set up the curriculum. In actual teaching, HSK test is one of the requirements for international students to graduate, which highlights the relationship between Chinese language teaching and HSK test. To solve this problem, we need to innovate between teaching methods, teaching language points and HSK interpretation, properly explore the curriculum of “promoting learning by examination, promoting teaching by examination, and combining examination with teaching”, and enhance the innovation and attraction of HSK curriculum to meet the actual needs of students. (3) Lack of characteristics of international students' vocational education for the talent training of international students, many teachers in higher vocational colleges have misunderstandings, especially professional teachers. On the one hand, it ignores the vocational education attribute of international students' training, separates the training of international students from the vocational and technical skills, and despises the professional skills teaching of international students, which leads to the cognitive deviation of the technical skills needs of international students; On the other hand, vocational Chinese textbooks lack the characteristics of higher vocational education, are not highly integrated with majors, and are not matched with teaching objects. Therefore, the training and curriculum setting of international students in higher vocational colleges should not only converge with Chinese students, but also teach students according to their aptitude to form a highly integrated and distinctive curriculum system for international students. In addition, we should also promote the exploration and innovation of teaching methods for international students in higher vocational colleges, especially in the practice of professional Chinese and professional scene Chinese. For example, explore and promote “project-based” or “scenario-based” Chinese teaching methods to improve the technical practice effect of international students training in vocational colleges. After several years of exploration and practice, the teaching of Chinese as a foreign language in the context of “Chinese+" has achieved some experience and results, but how to further improve the teaching content of “Chinese+" and build a more scientific and reasonable curriculum system still needs to be further considered and summarized in practice. The advantages of international Chinese education and vocational education should be fully considered, and the teaching content and teaching methods should always be set according to the needs of learners, industry enterprises and regional economic development. At the same time, we should adhere to the employment-oriented principle and organically combine the communicative and practical nature of language teaching with the professional and practical nature of skill teaching. In addition, in the reform of “three education”, teachers are fundamental. To change the current situation of traditional language teachers' lack of professional skills and the relatively weak language ability of professional teachers, and to cultivate the “Chinese+" teachers with both language teaching ability and practical skills is the key to promote the rapid development of “Chinese+". The teaching quality evaluation of international Chinese course in higher vocational colleges is affirmed as MAGDM. In this section, a numerical example for teaching quality evaluation of international Chinese course in higher vocational colleges is provided through PHF-TODIM-EDAS. There are five higher vocational colleges $VL_{i}\left(i=1,2,3,4,5\right)$ to be selected and six attributes are used to assess the teaching quality evaluation of international Chinese course of five higher vocational colleges (See Table 1):

Step 1 Build the PHFN-matrix $VH={\left[vh_{ij}\left(vp\right)\right]}_{5\times 6}$ in Table 2.

Step 2 Standardize the $VH={\left[vh_{ij}\left(vp\right)\right]}_{5\times 6}$ into $NVH={\left[nvh_{ij}\left(nvp\right)\right]}_{5\times 6}$ in Table 3.

**Table 3:** The $NVH={\left[nvh_{ij}\left(nvp\right)\right]}_{5\times 6}$

	VT_1_	VT_2_
$VL_{1}$	(0.32 (0.2), 0.38 (0.3), 0.47 (0.5))	(0.16 (0.2), 0.26 (0.3), 0.41 (0.5))
$VL_{2}$	(0.25 (0.0), 0.25 (0.3), 0.39 (0.7))	(0.14 (0.2), 0.29 (0.5), 0.49 (0.3))
$VL_{3}$	(0.32 (0.0), 0.32 (0.5), 0.38 (0.5))	(0.24 (0.0), 0.24 (0.5), 0.45 (0.5))
$VL_{4}$	(0.68 (0.0), 0.68 (0.7), 0.79 (0.3))	(0.76 (0.0), 0.76 (0.0), 0.76 (1.0))
$VL_{5}$	(0.28 (0.5), 0.32 (0.2), 0.46 (0.3))	(0.37 (0.5), 0.28 (0.2), 0.15 (0.3))
	**VT**_**3**_	**VT**_**4**_
$VL_{1}$	(0.49 (0.0), 0.49 (0.0), 0.49 (1.0))	(0.37 (0.0), 0.37 (0.3), 0.76 (0.7))
$VL_{2}$	(0.21 (0.3), 0.26(0.2), 0.37 (0.5))	(0.13 (0.3), 0.26 (0.5), 0.31 (0.2))
$VL_{3}$	(0.19 (0.0), 0.19 (0.5), 0.58 (0.5))	(0.17 (0.2), 0.25 (0.5), 0.42 (0.3))
$VL_{4}$	(0.54 (0.0), 0.54 (0.3), 0.76 (0.7))	(0.58 (0.0), 0.58 (0.5), 0.61 (0.5))
$VL_{5}$	(0.29 (0.0), 0.29 (0.5), 0.36 (0.5))	(0.32 (0.0), 0.32 (0.0), 0.32 (1.0))
	**VT**_**5**_	**VT**_**6**_
$VL_{1}$	(0.29 (0.0), 0.29 (0.7), 0.34 (0.3))	(0.34 (0.3), 0.17 (0.5), 0.47 (0.2))
$VL_{2}$	(0.24 (0.0), 0.24 (0.5), 0.41 (0.5))	(0.29 (0.0), 0.29 (0.5), 0.32 (0.5))
$VL_{3}$	(0.47 (0.0), 0.47 (0.0), 0.47 (1.0))	(0.19 (0.0), 0.19 (0.7), 0.36 (0.3)
$VL_{4}$	(0.67 (0.0), 0.67 (0.2), 0.78 (0.8))	(0.56 (0.0), 0.56 (0.2), 0.64 (0.8))
$VL_{5}$	(0.32(0.5), 0.34 (0.2), 0.43 (0.3))	(0.18 (0.3), 0.23 (0.5), 0.36 (0.2))

Step 3 Manage the weight numbers:

$$\begin{array}{l} vw_{1}=0.1707,vw_{2}=0.2028,vw_{3}=0.2194\\ vw_{4}=0.1261,vw_{5}=0.1355,vw_{6}=0.1455 \end{array}\text{.}$$

Step 4 Manage the relative weight numbers:

rvw=(0.7780,0.9243,1.0000,0.5747,0.6176,0.6632).

Step 5 Manage the $PHFNDD={\left(PHFNDD_{ij}\right)}_{5\times 6}$ (See Table 4):

**Table 4:** The $PHFEDD={\left(PHFEDD_{ij}\right)}_{5\times 6}$

	VT_1_	VT_2_	VT_3_
$VL_{1}$	−1.9161	−1.8503	−2.1036
$VL_{2}$	1.9286	1.2853	−1.1690
$VL_{3}$	−0.7274	−1.6775	−6.6466
$VL_{4}$	2.0059	−0.8981	2.4227
$VL_{5}$	−2.6178	−2.5276	−1.7742
	VT_4_	VT_5_	VT_6_
$VL_{1}$	−0.6901	−0.4100	3.0720
$VL_{2}$	0.5206	1.0871	2.3981
$VL_{3}$	−0.4812	1.9452	−2.2468
$VL_{4}$	2.5609	1.4018	1.0459
$VL_{5}$	−2.2314	−1.6383	−2.8390

Step 6 Construct the PHFNAS (See Table 5).

**Table 5:** The PHFNAS.

	VT_1_	VT_2_	VT_3_
PHFNAS	0.5088	0.3656	0.5284
	VT_1_	VT_2_	VT_3_
PHFNAS	0.4522	0.5903	0.5287

Step 7 Construct the PHFNPDA and PHFNNDA (See Table 6, Table 7):

**Table 6:** The PHFNPDA.

	VT_1_	VT_2_	VT_3_
$VL_{1}$	0.0000	0.0000	0.0000
$VL_{2}$	0.4745	0.6344	0.0755
$VL_{3}$	0.0000	0.0000	0.0000
$VL_{4}$	0.4912	0.0618	0.4716
$VL_{5}$	0.0000	0.0000	0.0088
	VT_4_	VT_5_	VT_6_
$VL_{1}$	0.0000	0.0000	0.4713
$VL_{2}$	0.1220	0.1702	0.3573
$VL_{3}$	0.0000	0.4097	0.0000
$VL_{4}$	0.5478	0.2580	0.1285
$VL_{5}$	0.0000	0.0000	0.0000

**Table 7:** The PHFNNDA.

	VT_1_	VT_2_	VT_3_
$VL_{1}$	0.3570	0.1880	0.0275
$VL_{2}$	0.0000	0.0000	0.0000
$VL_{3}$	0.0999	0.1426	0.5284
$VL_{4}$	0.0000	0.0000	0.0000
$VL_{5}$	0.5088	0.3656	0.0000
	VT_4_	VT_5_	VT_6_
$VL_{1}$	0.1306	0.2476	0.0000
$VL_{2}$	0.0000	0.0000	0.0000
$VL_{3}$	0.0870	0.0000	0.4285
$VL_{4}$	0.0000	0.0000	0.0000
$VL_{5}$	0.4522	0.5903	0.5287

Step 8 Construct the PHFNSP and PHFNSN (See Table 8).

**Table 8:** The PHFNSP and PHFNSN.

	PHFNSP	PHFNSN
$VL_{1}$	0.0686	0.1216
$VL_{2}$	0.3167	0.0000
$VL_{3}$	0.0555	0.1729
$VL_{4}$	0.3226	0.0000
$VL_{5}$	0.0019	0.2180

Step 9 Construct the PHFNNSP and PHFNNSN is in Table 9.

**Table 9:** The PHFNNSP and PHFNNSN.

	PHFNNSP	PHFNNSN
$VL_{1}$	0.2126	0.4424
$VL_{2}$	0.9817	1.0000
$VL_{3}$	0.1721	0.2070
$VL_{4}$	1.0000	1.0000
$VL_{5}$	0.0060	0.0000

Step 10 Construct the PHFNAV (See Table 10).

**Table 10:** The PHFNAV.

	PHFNAV	Order
$VL_{1}$	0.1406	3
$VL_{2}$	0.6492	2
$VL_{3}$	0.1138	4
$VL_{4}$	0.6613	1
$VL_{5}$	0.0040	5

Step 11 In line with the PHFNAV, the order is: $VA_{4}>VA_{2}>VA_{1}>VA_{3}>VA_{5}$ and $VA_{4}$ is the best higher vocational colleges.

**Table 1:** The six attributes for teaching quality evaluation of international Chinese course.

Attributes	Description
VT_1_	Classroom teaching preparation for international Chinese course
VT_2_	Classroom teaching process for international Chinese course
VT_3_	Teacher's reflection for international Chinese course
VT_4_	Teaching contents for international Chinese course
VT_5_	Student feedback for international Chinese course
VT_6_	Teaching techniques for international Chinese course

Then, PHF-TODIM-EDAS technique is constructed to cope with the college physical education teaching effect evaluation with CRITIC technique.

**Table 2:** The $VH={\left[vh_{ij}\left(vp\right)\right]}_{5\times 6}$

	VT_1_	VT_2_
$VL_{1}$	(0.32 (0.2), 0.38 (0.3), 0.47 (0.5))	(0.41 (0.5), 0.16 (0.2), 0.26 (0.3))
$VL_{2}$	(0.39 (0.7), 0.25 (0.3))	(0.14 (0.2), 0.29 (0.5), 0.49 (0.3))
$VL_{3}$	(0.32 (0.5), 0.38 (0.5))	(0.45 (0.5), 0.24 (0.5))
$VL_{4}$	(0.68 (0.7), 0.79 (0.3))	(0.76 (1))
$VL_{5}$	(0.32 (0.2), 0.46 (0.3), 0.28 (0.5))	(0.37 (0.5), 0.28 (0.2), 0.15 (0.3))
	**VT**_**3**_	**VT**_**4**_
$VL_{1}$	(0.49 (1))	(0.76 (0.7), 0.37 (0.3))
$VL_{2}$	(0.26(0.2), 0.37 (0.5), 0.21 (0.3))	(0.31 (0.2), 0.26 (0.5), 0.13 (0.3))
$VL_{3}$	(0.58 (0.5), 0.19 (0.5))	(0.17 (0.2), 0.25 (0.5), 0.42 (0.3))
$VL_{4}$	(0.76 (0.7), 0.54 (0.3))	(0.61 (0.5), 0.58 (0.5))
$VL_{5}$	(0.36 (0.5), 0.29 (0.5))	(0.32 (1))
	**VT**_**5**_	**VT**_**6**_
$VL_{1}$	(0.29 (0.7), 0.34 (0.3))	(0.47 (0.2), 0.34 (0.3), 0.17 (0.5))
$VL_{2}$	(0.41 (0.5), 0.24 (0.5))	(0.29 (0.5), 0.32 (0.5))
$VL_{3}$	(0.47 (1))	(0.19 (0.7), 0.36 (0.3)
$VL_{4}$	(0.67 (0.2), 0.78 (0.8))	(0.56 (0.2), 0.64 (0.8))
$VL_{5}$	(0.34 (0.2), 0.32(0.5), 0.43 (0.3))	(0.23 (0.5), 0.36 (0.2), 0.18 (0.3))

### 4.2 Sensitivity analysis

In this section, sensitivity analysis is implemented to verify the influence of parameter vθ on the final results of the PHF-TODIM-EDAS technique under PHFSs. The proposed PHF-TODIM-EDAS technique is implemented which considering two kinds of rational behaviors of DMs (risk aversion and risk seeking). Therefore, risk factor is depicted through employing vθ to implement DMs’ attitude towards risk aversion and risk seeking in real-life MADM. While vθ implements different attitudes of DMs towards risk aversion and risk seeking and it is implemented to have value between 1 and 2.5 in Ref. [57]. The sensitivity analysis is implemented in Table 11.

**Table 11:** The PHFNAV for different vθ

vθ	VL_1_	VL_2_	VL_3_	VL_4_	VL_5_
vθ=1.0	0.1406	0.6492	0.1138	0.6613	0.0040
vθ=1.2	0.1434	0.6619	0.1160	0.6743	0.0041
vθ=1.4	0.1462	0.6749	0.1183	0.6875	0.0042
vθ=1.6	0.1490	0.6881	0.1206	0.7010	0.0042
vθ=1.8	0.1520	0.7016	0.1230	0.7147	0.0043
vθ=2.0	0.1549	0.7154	0.1254	0.7287	0.0044
vθ=2.2	0.1580	0.7294	0.1279	0.7430	0.0045
vθ=2.4	0.1611	0.7437	0.1304	0.7575	0.0046
vθ=2.5	0.1642	0.7583	0.1329	0.7724	0.0047

In order to visualize the influence for different vθ values on the final ranking results, the final ranking results are implemented in Fig. 2. The final ranking results show that the psychological behavior of DMs effects the order slightly.

**Fig. 2:** The PHFNAV for different vθ

### 4.3 Comparative analysis

In this section, the PHF-TODIM-EDAS technique is compared with the PHFWA operator [38], PHFWG operator [38], PHF-TOPSIS technique [58], PHF-COPRAS technique [59], PHF-TODIM technique [60] and PHF-TODIM-PROMETHEE II technique [61], The final ranking results are constructed in Table 12 and Fig. 3.

**Table 12:** The order of different techniques.

Technique	The order
PHFWA technique [38]	$VA_{4}>VA_{2}>VA_{1}>VA_{3}>VA_{5}$
PHFWG technique [38]	$VA_{4}>VA_{2}>VA_{3}>VA_{1}>VA_{5}$
PHF-TOPSIS technique [58]	$VA_{4}>VA_{2}>VA_{1}>VA_{3}>VA_{5}$
PHF-COPRAS technique [59]	$VA_{4}>VA_{2}>VA_{1}>VA_{3}>VA_{5}$
PHF-TODIM technique [60]	$VA_{4}>VA_{2}>VA_{1}>VA_{3}>VA_{5}$
PHF-TODIM-PROMETHEE II technique [61]	$VA_{4}>VA_{2}>VA_{1}>VA_{3}>VA_{5}$
PHF-TODIM-EDAS technique	$VA_{4}>VA_{2}>VA_{1}>VA_{3}>VA_{5}$

**Fig. 3:** The order of different techniques.

Thus, From Table 12, Table 13, it is evident that the order of these techniques is slightly different, but these techniques have same higher vocational colleges and worst higher vocational college. This verifies the PHF-TODIM-EDAS technique is reasonable and effective. Thus, the main advantages of the proposed PHF-TODIM-EDAS technique are outlined: (1) the proposed PHF-TODIM-EDAS technique not only handles the bounded rationality in real MADM issues, but also portrays the hamming distances from the PHFNAS. (2) the proposed PHF-TODIM-EDAS technique analyze the behavior of the TODIM technique and EDAS technique as MADM when they are hybridized. The main disadvantages of the proposed PHF-TODIM-EDAS technique fails to manage the consensus theory and regret theory in the proposed MAGDM.

**Table 13:** WS coefficient calculation.

	PHF-TODIM-EDAS technique	PHFWA technique	PHFWG technique	PHF-TOPSIS technique
$VL_{1}$	4	4	4	4
$VL_{2}$	2	2	2	2
$VL_{3}$	1	1	3	1
$VL_{4}$	3	3	1	3
$VL_{5}$	5	5	5	5
Coefficients	WS	1.0000	0.7389	1.0000
	PHF-TODIM-EDAS technique	PHF-COPRAS technique	PHF-TODIM technique	PHF-TODIM-PROMETHEE II technique
$VL_{1}$	4	4	4	4
$VL_{2}$	2	2	2	2
$VL_{3}$	1	1	1	1
$VL_{4}$	3	3	3	3
$VL_{5}$	5	5	5	5
Coefficients	WS	1.0000	1.0000	1.0000

## 5 Conclusions

According to the 2019 Annual Report on the Quality of China's Higher Vocational Education, the number of full-time foreign students in higher vocational colleges reached 17,000, and more than 300 higher vocational colleges enrolled full-time foreign students in China. The talent training of international students has become an important part of the international running of higher vocational colleges and plays an important role in the process of implementing the reform of vocational education. At the same time, carrying out international student education is also one of the most direct and effective ways for higher vocational colleges to cultivate high-quality technical talents with an international perspective and serve the “the Belt and Road”. However, there are still significant differences between the teaching of Chinese for international students in higher vocational colleges and the teaching of Chinese in undergraduate colleges. The curriculum system, teaching mode, teaching material construction, teaching staff and other aspects are still in the initial exploration stage. Therefore, how to formulate a scientific and effective Chinese curriculum system for international students in higher vocational colleges is of great significance to improve the quality of international student talent training and promote the internationalization of higher vocational colleges. The teaching quality evaluation of international Chinese course in higher vocational colleges can be regarded as a MAGDM. Recently, the TODIM and EDAS technique has been employed to manage MAGDM. The PHFSs are employed as a useful tool for depicting uncertain information during the teaching quality evaluation of international Chinese course in higher vocational colleges. In this paper, the PHF-TODIM-EDAS technique is built to manage the MAGDM under PHFSs. At last, the numerical example for teaching quality evaluation of international Chinese course in higher vocational colleges is employed to show the PHF-TODIM-EDAS technique. The main contribution of this paper is constructed: (1) the TODIM technique based on EDAS technique has been extended to PHFSs based on CRITIC technique; (2) the CRITIC technique is employed to derive weight numbers under PHFSs. (3) the PHF-TODIM-EDAS technique is founded to manage the MAGDM under PHFSs; (4) a numerical case study for teaching quality evaluation of international Chinese course in higher vocational colleges and some comparative analysis is supplied to validate the proposed PHF-TODIM-EDAS technique.

There may be some possible limitations of this research for teaching quality evaluation of international Chinese course in higher vocational colleges, which can be further explored in future research: (1) It is a worthwhile research topic to apply prospect theory to teaching quality evaluation of international Chinese course in higher vocational colleges in the PHFSs environment [[62], [63], [64]]; (2) It is also worthwhile to apply regret theory to the study of teaching quality evaluation of international Chinese course in higher vocational colleges under PHFSs environment [[65], [66], [67], [68], [69]]; (3) In subsequent studies, the application of PHFSs needs to be investigated with consensus information measures for teaching quality evaluation of international Chinese course in higher vocational colleges [[70], [71], [72], [73], [74], [75]].

## Ethics declaration statement

The authors state that this is their original work, and it is neither submitted nor under consideration in any other journal simultaneously.

## Data availability

The authors agree that the data used in this manuscript is available to everyone and anyone can use this data by just citing this article.

## Funding information

This work was supported by the General Research Projects of Zhejiang Provincial Department of Education in 2023 (Project No.: 2023JYTYB11).

## CRediT authorship contribution statement

**Fangfang Xia:** Writing – original draft, Methodology, Data curation.

## Declaration of competing interest

The authors declare that they have no known competing financial interests or personal relationships that could have appeared to influence the work reported in this paper.
